# Bioactivity and Chemical Characterization of Sudanese Bee Honey: Crude Acacia and Its Organic Extracts

**DOI:** 10.1155/2022/8441239

**Published:** 2022-08-17

**Authors:** Mahasin Wadi

**Affiliations:** Department of Medical-Surgical, College of Nursing, Princess Nourah Bint Abdulrahman University, Riyadh, Saudi Arabia

## Abstract

Honey has recently been rediscovered as an antibacterial and wound-healing natural product. The medicinal properties of honey originate from the floral source used by bees. The objective of the current study was to evaluate the antimicrobial activity of Sudanese crude acacia bee honey and its solvent extracts regarding its biological activity and chemical characterization. To verify the nature of the antibacterial agent(s) of honey, sample (A) Sudanese crude unprocessed acacia bee honey obtained from west of Sudan (Nyala) during October 2019 was tested *in vitro* for antibacterial activity against 10 standard microorganisms *Enterobacter aerogenes*: ATCC: 13048, *Enterococcus faecalis*: ATCC: 29212, *Escherichia coli*: ATCC: 25922, *Klebsiella pneumoniae*: ATCC: 700603, *Pseudomonas aeruginosa*: ATCC: 27853, *Serratia marcescens*: ATCC: 8100, *Staphylococcus aureus*: ATCC: 29213, *Staphylococcus epidermidis*: ATCC: 12228, *Staphylococcus Methicillin* Sensitive MSSA: ATCC: 29213, and *Staphylococcus Methicillin-*Resistant MRSA: ATCC: 23591. Extraction of honey sample was carried out by petroleum ether followed by ethyl acetate using liquid/liquid extraction technique, using separating funnels. All organic extracts in addition to their aqueous residue were tested *in vitro* for antibacterial activity against the10 standard microorganisms. Ethyl acetate extract was subjected to gas chromatography-mass spectrometer (GC-MS) for chemical characterization. Sudanese crude unprocessed acacia honey showed inhibitory effects against the 10 standard microorganisms. Petroleum ether extract showed no antibacterial activity against the tested organisms, while its water residue exhibited remarkable activity. The ethyl acetate extract exhibited strong antibacterial activity against the tested organisms, while its aqueous residue showed no activity. Ethyl acetate extract subjected to gas chromatography-mass spectrometer (GC-MS) showed twenty-one chemical constituents. The GC-MS showed twenty-one chemical compounds, and phenolic compound was the highest concentration. Ethyl acetate extract exhibited strong antibacterial activity which can be formulated as topical dressing for wounds and burns. The usage of honey in a professional context should be taken into consideration while treating burns and wounds.

## 1. Introduction

Apitherapy has become the alternative medicine for treating certain diseases and chronic wounds not responding to conventional treatment. The antibacterial properties of honey have long been recognized, with a wide range of potential against bacteria and other pathogens. Its antibacterial effectiveness is influenced by a number of crucial parameters, such as osmolarity, H_2_ O_2_ content, low pH, phenolic acid concentrations, and flavonoids [1]. Honey was widely used in herbal medicine all over the world. Variation in chemical and phytochemical properties of honey was attributed to floral origin. Honey was discovered to induce the release of a number of cytokines, including tumor necrosis factor, a protein that decreases tissue inflammation and stimulates white blood cells, both of which are essential for healing [1]. Honey is accountable for all of its biological activities, mainly to its composition [2]. Honey is made up of several different chemicals. Sugars, bee proteins, vitamins, minerals, and polyphenols are all found in honey, and polyphenols are the most effective antioxidants [3]. The biological activity of honey and its polyphenolic content are strongly correlated, and polyphenols are secondary plant metabolites that act as antioxidants in the body [3]. Gallic acid, catechins, epicatechins, chlorogenic acids, caffeic acids, coumaric acids, and quercetin are the most common polyphenols found in honey [4]. Antioxidant of honey potential is evaluated not only by the existence of total phenolic compounds, but also by the presence of flavonoids, which play a key role in the oxidative fermentation method [5]. Flavonoids are the most common phytochemicals found in honey, such as quercetin, kaempferol, luteolin, chrysin, pinobanksin, galangin, and pinocembrin [6]. Antibacterial activity of honey has been discovered after it was extracted and fractionated using organic solvents. Extraction of honey ethyl acetate and fractionation with organic solvents showed potent antibacterial activity [7]. The volatile fraction of honey has been investigated using a range of extraction methods combined with gas chromatographic (GC) analysis [8].

Volatile organic compounds (VOCs) are one of the most common secondary metabolites in the study of floral markers that can be used to assign honey to a particular botanical origin [9]. Polyphenols, especially flavonoids, phenolic acids, and their derivatives, are also present in honey [10]. Polyphenols and phenolic acids can be present in a number of plants, including nectar, pollen, honeydew, and propolis [11]. At low concentrations, the ethyl acetate fractions had antibacterial, anticandidal, and antifungal properties (12). The active fraction of honey was transformed into a semisolid dosage form. Honey extract release from various ointment bases was affected by the base constituents and stabilizers [12]. Honeys obtained from Danish flora have antibacterial properties, owing to a barrier effect of viscosity, osmolality, acidity, bioactive peptides, and, most notably, the presence of hydrogen peroxide [13]. Commercially available wound dressings include vegetable fibers, protective films, hydrogels, and hydrogels enriched with nitrogen oxides [14, 15]. Since ancient times, honey has been utilized for medical purposes either alone or in conjunction with other compounds. Honey is a heterogeneous material with antimicrobial and anti-inflammatory properties, as well as the ability to speed up the healing process after skin or peritoneal damage [16, 17]. The antibacterial effects of honey have been traced to a number of compounds [18–20].

Honey methanol extracts were found to have antibacterial efficacy across a wide variety of bacteria [21]. Honey has long been known to inhibit a wide variety of bacterial species. More than 60 bacterial species, including aerobes and anaerobes, have been demonstrated to be inhibited by honey, Gram positives, and Gram negatives [22]. A close correlation has been found between the content of phenolic compounds in different botanical honeys and their antioxidant and antibacterial properties [23, 24]. Flavonoids were detected in European Eucalyptus honeys using a typical and characteristic high-performance liquid chromatography (HPLC) profile [25]. The previous findings confirmed that the antibacterial properties of honey are primarily due to phenolic compounds, especially flavonoids and phenyl propanoids [26]. Thymus honey demonstrated the highest expected inhibition of all the bacteria strains tested in an antibacterial assay. The antibacterial activity of honey against *Escherichia coli*, *Staphylococcus aureus*, and *Bacillus subtilis* can mainly be affected by its phenolic content [27].

Honey has been used for medicinal purposes since ancient times, either alone or in conjunction with other compounds. Honey is a heterogeneous material with antimicrobial and anti-inflammatory properties, as well as the ability to accelerate up the healing process after skin or peritoneal damage [28, 29]. Honey contains high glycine, methionine, and proline, both of which are necessary for the production of collagen and fibroblast deposition, which are the two most important factors in wound healing [30]. Many essential organic compounds have been found in various types of honeys using GC-MS methods [31]. Gas-chromatography-Mass-spectrometer (GC-MS) study of three honey samples of well known floral origin: Each honey contained a number of volatile components, including liphatic and aromatic compounds, cyclic and monocyclic monoterpenes and other oxygenated derivatives, furan derivatives, sulfur, and nitrogen-containing compounds [32].

According to the results of GC-MS analysis of honey, a total of 41 aroma compounds were identified and quantified, including 11 acids, 5 alcohols, 5 aldehydes, 4 ketones, 3 terpenes, 3 lactones, 3 phenols, 3 esters, 3 pyrans, and 1 norisoprenoid [33].

Both raw honeys and their phenolic fractions showed antibacterial activities, and chestnut honeys showed the highest activities. These findings indicate that phenolic compounds, especially flavonoids and phenyl propanoids, are primarily responsible for antibacterial properties of honey [34]. Cinnamon bark and honey extract are indicated to have strong potential activity against acne causing bacteria and can therefore be used as topical antiacne preparations Honey with high phenolic content had high antioxidant and antibacterial activity [35]. Dark honey has been reported to be a potent antioxidant and antibacterial component [36]. The most effective bactericidal effect against *Helicobacter pylori* test isolates was obtained with 5% v/v (1/2 MIC) concentration of South African honey chloroform extract [37].

The phytochemical composition of honey affects its biological function, and the same compounds are commonly found to contain both antimicrobials and antioxidants [38]. Honey's phenolic composition is largely determined by its floral origin; in fact, it can be used to classify and authenticate honey, especially unifloral varieties [39]. Unifloral honeys derived from the respective plant sources should have a distinct pattern of phenolic compound distribution. Flavonoids in honey may originate from nectar, pollen, or propolis [40].

The active antibacterial substance(s) in honey was identified as “Inhibine.” The idea of “Inhibine” was related to the hydrogen peroxide present in honey due to the activity of glucose oxidase enzyme normally present in honey secreted from the bees' hypopharyngeal glands and glucose oxidase enzyme acting on honey glucose to generate hydrogen peroxide and oxygen [41].

The aim of the current study is to evaluate the antibacterial activity of Sudanese crude acacia bee honey and its extracts against 10 standard different bacteria, as well as to characterize its chemical composition according to the floral and geographic source.

## 2. Materials and Methods

### 2.1. Bee Honey Sample

Crude unprocessed a monofloral sample of Sudanese acacia bee honey sample (A) was collected from a local apiary, Nyala west of Sudan, during September 2019. Honey sample has been kept at room temperature in a sterile glass container. Honey sample was labeled according to the source, location, pH, date of collection, and floral origin. Honey sample was checked for sterility by conventional microbiological methods in Microbiology Laboratory.

### 2.2. Chemicals and Reagent

All chemicals and reagents were analytically grade purity.

### 2.3. Standard Organisms

The following 10 standard organisms Gram-positive, Gram-negative, Microbiology Reference Laboratories were obtained, the American Type Culture Collection (ATCC), 12301 Drive, Rockville, MD 20852, USA: *Enterobacter aerogenes (E. aerogenes)*: ATCC: 13048, *Enterococcus faecalis (E.faecalis)*: ATCC: 29212, *Escherichia coli (E.coli)*: ATCC: 25922, *Klebsiella pneumoniae (K. pneumoniae)* : ATCC: 700603, *Pseudomonas aeruginosa (P.aeruginosa)*: ATCC: 27853, *Serratia marcescens (S.marcescens)*: ATCC: 8100, *Staphylococcus aureus (S.aureus )*: ATCC: 29213, *Staphylococcus epidermidis (S.epidermidis)*: ATCC: 12228, *Staphylococcus Methicillin* Sensitive (MSSA): ATCC: 29213, and *Staphylococcus Methicillin*-Resistant (MRSA): ATCC: 23591 [42].

### 2.4. Inoculum Preparation

Pure culture and standard inoculum size must be maintained for antibacterial susceptibility. Control organisms were suspended in a sterile saline to match 0.5 McFarland standard tube, which is commercially available, and provide an optical density of 1.5 × 10^8^ colony-forming units (CFU/ml). The well plate technique was used for testing honey antibacterial activity due to its high viscosity [42]. .

### 2.5. Well Plate Technique

The technique of seeded agar diffusion was used [43]. Muller Hinton agar culture medium has been reconstituted and sterilized (using autoclave) at 121°C for 15 minutes and allowed to cool at 48°C and inoculated with 0.1 ml of standardized 24 broth culture of bacterial suspensions that match the turbidity of the 0.5 McFarland standard tube (1.5 × 10^8^) (FU/ml). The inoculated medium was distributed aseptically in 20 ml volumes into sterile Petri dishes (95 mm internal diameter) and allowed to set. The seeded agar plate that had solidified was then packed at 4°C until use. Four cups (8 mm diameter) were cut using 8-mm sterile cork borer, and the cut disc of agar was removed, and 0.2 ml of each honey sample was carefully added to diffuse. The seeded plates were incubated at 37°C for 18-24 hours [42]. The diameter of the resultant growth inhibition zone was measured in mm ± standard deviation (SD. Honey sample was tested for antibacterial activity against each organism in four replicate. The average diameter of the inhibition zone was measured.

### 2.6. Liquid–Liquid Extraction Procedure

#### 2.6.1. Honey Extractions

A 25 gm of honey sample was diluted with 25 ml distilled water to give 50% dilution. The diluted honey sample was extracted with 50 ml (5 × 10ml) of petroleum ether (60-80°C) using liquid/liquid extraction technique, using separating funnels. The upper phase petroleum ether (PE) was separated with anhydrous sodium sulfate and then concentrated under reduced pressure vacuum using Buchi Rota evaporator. 10 ml of the concentrated extract was collected. The remaining water residue (lower phase) was further partitioned with 50 ml (5 × 10 ml) ethyl acetate using separating funnel. The upper organic phase (ethyl acetate) was separated with anhydrous sodium sulfate, which was concentrated under reduced pressure to 10 ml [44].

### 2.7. *In Vitro* Antibacterial Activity of Crude Bee Honey and Honey Extracts

Crude Sudanese acacia bee honey sample was tested against 10 standard microorganisms in four replicates using well plate technique. Honey extracts petroleum ether and ethyl acetate extract in addition to their water residue (0.2) were assayed for antibacterial activity against the same 10 standard microorganisms using the same well plate technique under the same condition. The mean of inhibition zone diameter was tabulated. Petroleum ether and ethyl acetate solvents were checked for their antibacterial activity by conventional microbiological methods.

### 2.8. Gas Chromatography Mass Spectrometer Preparation of Honey Sample

Honey ethyl acetate extract sample (A), was analyzed using GC-MS SHIMADZU-QP5050 GC-174, with electron impact detector, equipped with column RTX5M5 packed with 5% diphenyl-95% dimethylpolysiloxane. Length is 30 meter, interior diameter is 0.25 mm, film thickness is 0.25 *μ*m, and the gas carrier was helium, at 1 ml/min rate, with injection volume of 1 *μ*L. The injector and detector temperature were maintained at 50°C starting up to 280°C, respectively [45].

Honey ethyl acetate extract sample (A) was automatically injected. Electron impact mass spectra were recorded in 40-500 mass range. An electron ionization energy is 70 V. Started time is 2 minutes, and end time is 45 minutes. Software has been used to automatically record spectral data throughout the elution process. Identification was carried on the basis of beak development compared to mass spectra library.

## 3. Results

### 3.1. *1n Vitro* Antibacterial Activity of Sudanese Acacia Bee Honey

Unprocessed Sudanese acacia bee honey was tested for sterility at Microbiology Laboratory and was proved to be sterile without bacterial growth.

Sudanese acacia crude raw unprocessed bee honey obtained from Nyala west of Sudan was tested for antibacterial activity against 10 standard bacterial strains, Gram-positive and Gram-negative: *E. aerogenes*: ATCC: 13048, *E. faecalis*: ATCC: 29212, *E. coli*: ATCC: 25922. *K. pneumoniae*: ATCC: 700603, *P.aeruginosa*: ATCC: 27853, *S. marcescens*: ATCC: 8100, *S. aureus*: ATCC: 29213, *S. epidermidis*: ATCC: 12228, *Staphylococcus Methicillin* Sensitive MSSA: ATCC: 29213, and *Staphylococcus Methicillin*-Resistant MRSA: ATCC: 23591. Tested honey sample against 10 standard organisms indicated that it had inhibitory effects on both Gram-positive and Gram-negative organisms (Table 1). The following Gram-positive organisms, *S. aureus*, *S. aureus Methicillin-Resistant MRSA*, *and S. aureus Methicillin Sensitive MSSA*, were shown to be the most susceptible organisms to the tested honey (Table 1). The honey sample had very identical or equivalent inhibitory effects on Gram-negative species, as seen by the very small or no differences in growth inhibition zones (Table 1). The examined honey was proven to be effective against Gram-negative microorganisms, *Pseudomonas aeruginosa* which is the most resistant to common antibiotics, although *Klebsiella pneumoniae*, *Enterobacter aerogenes*, and *Serratia marcescens* demonstrated considerable sensitivity to the tested honey sample. Gram-negative species had inhibitory zones that were almost of identical inhibition one (Table 1).

### 3.2. Antibacterial Activity of Petroleum Ether, Ethyl Acetate Extracts, and Their Water Residue of Sudanese Acacia Bee Honey

Petroleum ether and ethyl acetate solvents tested for antibacterial activity showed no activity.

*In vitro* antibacterial activity of petroleum ether, ethyl acetate fractions, and their water residue were carried out against the same 10 standard organisms using well plate seeded agar diffusion technique. The petroleum ether extract tested against the 10 standard organisms showed no activity, while its water residue exhibited effective antibacterial activity (Table 1). The ethyl acetate extract exhibited strong antibacterial activity against the tested organisms (Table 1), while its water residue showed no activity.

### 3.3. Gas Chromatography Mass Spectrometer (GC-MS) Analysis of Sudanese Acacia Bee Honey

#### 3.3.1. GC-MS Chromatogram of Honey

The GC-MS analytical approach is the consequence of integrating two analytical techniques: capillary column GC, which separates the components of a mixture, and mass spectrometry (MS), providing the necessary details to determine the structure of component. The interpretation of the chromatograms is achieved using the “Data Analysis” program. The peaks eluted at short retention times were mostly volatile oxygenated compounds, while those eluted at long retention times were semivolatile compounds (Figure 1).

Component identification for the sample was achieved by comparison of their retention times and mass fragmentation patents with the ones available in the National Library Institute of Standards and Technology (NIST).

Gas chromatography-mass spectrometer (GC-MS) analysis of Sudanese acacia honey obtained from west of Sudan revealed 21 compounds. The most common volatile substances of Sudanese acacia honey identified are Urs-12-en-28-al, 3-(acetyloxy)-, (3.beta.)-, and Phenol, 2,4-bis(1,1-dimethylethyl)- (Table 2).

The volatile profile of Sudanese acacia honey obtained from west Sudan was demonstrated in Table 2. The highest concentration is the phenolic substance Phenol, 2,4-bis(1,1-dimethylethyl)- 13.64% and Urs-12-en-28-al, 3-(acetyloxy)-, (3.beta.) (Table 2).

## 4. Discussion

Understanding the composition of honey and how it varies depending on the floral source, age, and location of production is crucial to understanding its microbiological activity. No information has been available on the variation and composition of Sudanese honeys. Therefore, a systematic bioassay directed fractionation was deemed necessary.

Medicinal use of honey particularly as a topical antibacterial dressing has gained a significant interest in recent years. Honey has been used successfully to treat infections that have failed to respond to conventional antiseptic and antibiotic care.

The tested honey sample showed strong antibacterial activity against tested standard Gram-positive and Gram-negative organisms. The Gram positive showed remarkable sensitivity to tested honey samples. *Staphylococcus aureus* and Methicillin-resistant *Staphylococcus aureus* (MRSA) exhibited the highest sensitivity toward the tested honey sample inhibition zone (34 mm). Methicillin-resistant *Staphylococcus aureus* (MRSA) is a major public health issue that causes hospital and community-acquired infections all over the world. *S. aureus* is a Gram-positive bacterium that has been linked to skin diseases such impetigo, furuncles, boils, sties, pustules, burns, and wounds. Antibiotic-resistant *S*. *aureus* strains are the leading source of infections, particularly in hospitals settings [46]. Thus, honey can be used to treat various infection caused by *Staphylococcus aureus* (MRSA).

The Gram-negative organisms was much less sensitive to honey than the Gram-positive group. These findings support those of the earlier investigator who confirmed that honey has been reported to have an inhibitory effect to around 60 species of bacteria including aerobes and anaerobes, Gram positives, and Gram negatives [22]. Gram-negative bacteria *P. aeruginosa*, the most stubborn organism, was found responsive to the tested honey sample that was evaluated. This species is an important opportunistic pathogen intrinsically resistant to many antibiotics. *Pseudomonas* was regarded as a multidrug-resistant organism to the most widely used antibiotics, antiseptic, and disinfectant, and it was assessed as the important pathogen in chronic wounds and burns infection. It was also taken into consideration the most major infectious agent of hospital-acquired infection. Some strains of *P. aeruginosa* have been found to be resistant to nearly all or all antibiotics including aminoglycosides, cephalosporins, fluoroquinolones, and carbapenems [47]. A number of clinical trials have been published using honey against *Pseudomonas* infection. It was also noted that the susceptibility of Gram-negative bacteria to honey was attributed to the presence of hydrogen peroxide and potent antioxidants, as well as a naturally low pH that inhibits bacterial growth, and the abundance of phenolic acids, lysozyme, and flavonoids [48]. Thus, honey might be an appropriate therapeutic alternative to those antibiotics as in cases of hospital-acquired infections with *P. aeruginosa.*

Petroleum ether fraction of the bee honey sample showed no antibacterial activity against the tested standard microorganisms, while its aqueous residue showed an antibacterial activity. The ethyl acetate fraction tested against the 10 standard microorganisms exhibited strong antibacterial activity, while its water residue showed no activity. The absence of antibacterial active component in petroleum ether fraction and predominance of activity in the aqueous residue coupled with the total extractability of the active substance(s) with the ethyl acetate demonstrated the hydrophilic nature of the bioactive agent(s). The total removal of the bioactive agent(s) from the aqueous residue which is expected to contain most or all of the sugar and hydrogen peroxide makes these results perplexing in the contextual framework of the Inhibine's theory. These findings are consistent with previous research carried by Bogdanov who extracted and fractionated honey using organic solvents and ethyl acetate extract that revealed potent antibacterial activity [7]. Our present findings supported the previous study that reported the ethyl acetate fractions showing antibacterial, anticandidal, and antifungal effects at low concentration. [11, 12]. The present study confirmed that the antibacterial agent(s) can be extracted by organic solvent; this in line with previous report that honey methanol extracts resulted in a broad spectrum of antibacterial activity [21].

Honey contains a wide variety of phenolic compounds; phenolic acids and flavonoids are the two main classes of these compounds. The amount of phenolic compounds varies depending on the honey's flora and geographical origin. Honey's antibacterial activities are mostly due to phenolic chemicals, particularly flavonoids and phenyl propanoids [34]. Floral origin facilitates satisfactory discrimination between different types of honey; accordingly different honey colors ranging from white, golden to black honey were obtained. However, different aroma, taste, and pH can be obtained. Accordingly certain honey types are preferred. The presence of phenolic compounds in different botanical honeys and their antioxidant and antibacterial properties have been discovered to be closely related [23, 24].

The antibacterial activity of honey may be attributed to the phenol and flavonoids. These outcomes indicate that a component of antimicrobial effect might originate from plant rather than from the bees [3]. In the present study, ethyl acetate extracts of Sudanese acacia bee honey was subjected to GC-MS analysis which revealed 21 different compounds with high phenolic component. Phenolic compound was detected in sample (A), obtained from west Sudan, floral origin acacia. The findings of the current analysis showed that the phenolic compounds of honey may correlate with geographical and botanical origin. These compounds are known to have some biological activity such as antibacterial. The previous finding noted that honey flavonoids can be included in nectar, pollen, and propolis [40]. Our present study supported the previous research of using GC-MS methods, for many important organic compounds have been detected in different types of honeys [31]. The present findings showed that volatile extraction of honey sample has the highest concentration of phenolic substances, which is mainly attributed for antibacterial activity. The quality of honey is evaluated by its botanical or floral origin and chemical constituents [49]. In some honeys, such as those obtained from lavender and acacia, no specific phenolic components have been found as suitable floral markers [50]. Honey is acidic in nature, with gluconic acid being the most common acid produced by glucose oxidase in the presence of water and oxygen, as well as bacteria of the genus Gluconobacter, which are infrequently isolated from ripening nectar [51]. Sudanese acacia honey exhibited antibacterial activity against different Gram-positive and Gram-negative organisms. This result seems in consistent with the previous observations that monofloral honey has a greater antibacterial effect than multifloral honey [44]. There is a good correlation between total phenolic content and the biological activity of honey samples [52]. Alternative medicines have been regarded by the World Health Organization (WHO) as a low-cost option to achieving universal health coverage for the world's population, and member authorities have been encouraged to use plant-based alternative medicines rationally [53].

As the phenolic compound regarded the active component of the antibacterial activity of honey, the volatile profiles observed for the honey extractives were also highly consistent.

The present study confirmed that the active substance(s) in honey was extracted by ethyl acetate; this gives support to the belief that the antibacterial effect of honey might be due to phenolic compounds. Natural products is recently the focus of antifungal, antiviral, and antibacterial activity.

## 5. Conclusion

Natural crude unprocessed Sudanese acacia honey demonstrated a potent *in vitro* antibacterial activity against a large spectrum of Gram-positive and Gram-negative bacteria. Honey was found to be effective in inhibiting *P. aeruginosa* and MRSA. Honey ethyl acetate extract exhibited powerful antibacterial activity towards tested bacteria.

Most of the honey inhibitory effects was attributed to the phenolic substances as detected by and GC-MS analysis. This antibacterial capability could be attributed to the plant's wide range of bioactive phenolic components. The findings of the present study confirmed that the bactericidal effect of honey could be attributed to agent(s) that was extracted using ethyl acetate solvent; it is not related to its high sugar content or hydrogen peroxide formation. Honey derived from a variety of botanic sources has high antimicrobial activity. Possibility the application of this natural product to clinical practice for treatment infections will be the focus of extensive research in the near future. Sudanese acacia honey are characterized and classified according to the geographical diversity.

## Figures and Tables

**Figure 1:** Eluted components of ethyl acetate extract of Sudanese acacia bee honey using GC-MS.

**Table 1:** Antibacterial activity of Sudanese acacia bee honey sample, petroleum ether, ethyl acetate extract, and their water residue against 10 standard organisms.

Bacterial strains	*E. faecalis*	*S. aureus*	*S. epidermidis*	MSSA	MRSA	*E. coli*	*E. aerogenes*	*P. aeruginosa*	*K. aerogenes*	*S. marcescens*
Diameter of growth inhibition zones in mm ± (SD)										
Crude honey sample A	26 ± (1)	34 ± (1)	32 ± (1)	32 ± (1)	34 ± (1)	27 ± (0.8)	26 ± (0.8)	25 ± (0.5)	25 ± (0.5)	25 ± (0.5)
Petroleum ether extract	0	0	0	0	0	0	0	0	0	0
Water residue	20 ± (0.5)	23 ± (0.5)	20 ± (0.5)	20 ± (0.5)	24 ± (0.5)	22 ± (0.5)	20 ± (0.5)	20 ± (0.5)	22 (0.5	20 ± (0.5)
Ethyl acetate extract	19 ± (0.7)	19 ± (0.7)	18 ± (0.4)	18 ± (0.4)	20 ± (0.5)	20 ± (0.5)	18 ± (0.5)	21 ± (0.6)	18 ± (0.5)	18 ± (0.5)
Water residue	0	0	0	0	0	0	0	0	0	0

**Table 2:** Identification of chemical compounds of Sudanese acacia honey using GC-MS.

ID#	Name	Ret. time	Area	Area%
1.	1-Dodecene	7.080	225123	0.50
2.	Dodecane	7.193	76025	0.17
3.	1-Tetradecene	9.942	1027666	2.27
4.	Phenol, 2,4-bis(1,1-dimethylethyl)-	11.730	6183896	13.64
5.	1-Heptadecene	12.555	3893000	8.59
6.	Hexadecane	12.636	375677	0.83
7.	1-Nonadecene	14.916	4090331	9.02
8.	Behenic alcohol	17.055	3320596	7.33
9.	1-Heptacosanol	19.005	2364947	5.22
10.	Pentacosane	19.956	420927	0.93
11.	[1,1′-biphenyl]-2,3′-diol, 3,4′,5,6′-tetrakis(1,1-dimethylethyl)-	20.616	336858	0.74
12.	n-Tetracosanol-1	20.793	1825876	4.03
13.	Gamma-sitosterol	20.997	1515652	3.34
14.	Octacosane	21.666	1427451	3.15
15.	Beta-sitosterol acetate	21.967	2340144	5.16
16.	1-Eicosene	22.444	1126937	2.49
17.	Eicosane	23.249	1732880	3.82
18.	Urs-12-en-28-al, 3-(acetyloxy)-, (3.beta.)-	25.979	6375494	14.05
19.	Nonanoic acid, phenylmethyl ester	26.285	3026969	6.68
20.	Tetratriacontane	26.589	736957	1.63
21.	Gitoxigenin	28.532	2907578	6.41

## Data Availability

The data sets used and analyzed in the current study are included in the article.
